The article "Post-mortem analysis of neuroinflammatory changes in human Alzheimer’s disease" was published in 2015. Journal: Alzheimers Res Ther.

# Post-mortem analysis of neuroinflammatory changes in human Alzheimer’s disease

**DOI:** 10.1186/s13195-015-0126-1

**Published:** 2015-04-22

**Authors:** Diego Gomez-Nicola, Delphine Boche

**Affiliations:** Centre for Biological Sciences, Faculty of Natural and Environmental Sciences, University of Southampton, Southampton General Hospital, Tremona Road, Southampton, SO16 6YD UK; Clinical Neurosciences, Clinical and Experimental Sciences, Faculty of Medicine, University of Southampton, Southampton General Hospital, Tremona Road, Southampton, SO16 6YD UK

## Abstract

Since the genome-wide association studies in Alzheimer’s disease have highlighted inflammation as a driver of the disease rather than a consequence of the ongoing neurodegeneration, numerous studies have been performed to identify specific immune profiles associated with healthy, ageing, or diseased brain. However, these studies have been performed mainly in *in vitro* or animal models, which recapitulate only some aspects of the pathophysiology of human Alzheimer’s disease. In this review, we discuss the availability of human *post-mortem* tissue through brain banks, the limitations associated with its use, the technical tools available, and the neuroimmune aspects to explore in order to validate in the human brain the experimental observations arising from animal models.

## Introduction

The concept of research on human samples has been pioneered by neuropathologists who had an interest in research and who started to archive brain specimens referred for diagnosis, such as the one developed by John Corsellis in 1950 [1]. Development of novel technologies to detect biological molecules and increased collaboration with scientists highlights the need for the use of human samples, especially in the neurosciences. Indeed, one of the major limitations to our knowledge of human neurological diseases resides partly in the limits inherent to animal models, which mimic some aspects of the human neurological disorder without reproducing its complexity arising from both genetic and environmental factors. For example, more than 50 different animal models have been generated to explore Alzheimer’s disease (AD) [2] and more than 20 models are available for the study of schizophrenia [3] without clear consensus about the similarities with human disease. The underuse of *post-mortem* human brain tissue also impedes the deeper understanding of the pathophysiological processes ongoing in the diseased brain [3].

Therefore, in the mid-20th century, the notion of brain banking to archive, collect, and use human brain samples became essential with the aim to facilitate access to the tissue, to simplify the administrative burden for the researcher, and to improve their quality for cutting-edge research on neurological diseases. In this review, we discuss the pros and cons related to the use of human tissue, the parameters susceptible to influence the neuroinflammatory changes, and how to analyse them in AD.

The article "Post-mortem analysis of neuroinflammatory changes in human Alzheimer’s disease" was published in 2015. Journal: Alzheimers Res Ther.

## Requirements and limitations to the use of *post-mortem* brain tissue

### Ethics

Networks of brain tissue banks have been created to allow request of tissue through a unique portal such as the consortium BrainNet Europe in 2001 under the European Commission or the UK Network of Brain Tissue Banks in 2009 by the Medical Research Council. In the UK, the use of human tissue is regulated by the Human Tissue Authority (HTA) and brain banks are licensed to operate as research tissue banks by the HTA under ethical approval provided by an ethics committee. This implies that the use of human tissue for a specific project is subject to approval by the brain bank committee. This is a compulsory step that could hinder the researcher and thus might appear as a limitation. However, under the approval of the brain bank, the study is ethically covered by the bank, saving administrative burden to the researcher and thus optimising the time spent on the project. This procedure is not restricted to the UK; the same principle applies worldwide [4]. Information about US brain banks is found under the platform National Institutes of Health NeuroBioBank. The Australian Brain Bank Network, in addition to provide tissue for research, offers a neuropathology diagnostic service and education and training opportunities. Asia has started to set up brain banks in Japan, India, and China. Two brain banks are also present in South America: one in Brazil (the Brain Bank of the Brazilian Aging Brain Study Group, Sao Paulo) and one in Argentina.

### Quality of the tissue

Quality of the tissue during its acquisition and long-term preservation is the principal objective of the bank. Different parameters may impact on the integrity of the tissue and thus on any biological molecules. Therefore, it is important to take into account these factors in the analysis of inflammatory events. These include age (the immune profile is known to evolve with ageing [5]), gender, genetic heterogeneity, agonal status (defined as the deep infrequent respiration in the final moments before death), preterminal medication, cause of death, concomitant disease, *post-mortem* interval [6], and time in the fixative. In addition, the potential role of systemic inflammatory diseases and infections may influence the cerebral inflammatory status [7]. Clinical studies have reported an accelerated deterioration of the cognition in the AD patients affected by systemic infections [8,9], and experimental studies demonstrated that systemic infection can switch the brain inflammation to a more aggressive phenotype, resulting in increased neurodegeneration [10,11].

The article "Post-mortem analysis of neuroinflammatory changes in human Alzheimer’s disease" was published in 2015. Journal: Alzheimers Res Ther.

It is usual practise in most of the prospective brain banks to fix one hemisphere and freeze the other hemisphere when collecting tissue. The preparation of the fixed tissue is a routine procedure used for diagnosis in any pathology department and thus a standardised protocol among the brain banks. Fixed tissue is used for histological staining and protein detection by immunohistochemistry, and the main difficulty is to achieve optimal specificity of the staining. Indeed, optimisation of the staining might require testing antibodies from different companies, using several pre-treatments (that is, antigen retrieval), and importantly ensuring that the detected staining is specific. This could be tested by using samples from another organ that expresses the protein of interest (such as the lymph node for any macrophage/microglia proteins) or by a blocking experiment to test the specificity of the primary antibody or by doing both [12]. The preparation of fresh frozen tissue is more challenging as genetic material is susceptible to degradation under the factors described above and sometimes is not available from the archives of tissue banks. In addition, the development of genomic and proteomic technologies has highlighted the importance of obtaining high-quality RNA. If available, brain tissue pH and RIN (RNA integrity number) value are proxy indices of agonal status [13] and thus good indicators of the quality of the frozen tissue as far as the preservation of RNA and proteins is concerned [14]. Proteins are known to be more resistant as they can still be detected in tissue even when RNA is degraded [14]. Overall, standardized protocols have been developed and optimized by brain banks to minimize the impacts of *pre*- and *post-mortem* conditions.

## Information required for the analysis of the immune response in Alzheimer’s disease

To ensure that the detection of the inflammatory profile is optimal in the human samples, the study should be adequately designed to overcome or minimize the impact of the factors discussed above. This can be achieved by the following:

- Age and gender: to match selected cases.
- Genetic heterogeneity: to determine the sample size necessary to reach statistical power [15].
- Agonal status: to obtain pH and RIN values. The RIN algorithm has been designed to provide unambiguous assessment of RNA integrity based on a numbering system from 1 to 10, with 1 being the most degraded profile and 10 being the most intact [13]. The choice of the RIN value will depend on the technique to be used, as microarray analysis will need a higher RIN value than RT-PCR [14].
- Pre-terminal medication or concomitant disease or both: to get access to the *post-mortem* report and to control the quantitative analysis for these confounding factors.
- Cause of death: to refer to the death certificate.
- *Post-mortem* interval: to select cases with the shortest interval and usually no more than 72 hours.
- Time in the fixative: to ensure that sections are provided from blocks taken at the *post-mortem* examination after a standardised time in the fixative.

The article "Post-mortem analysis of neuroinflammatory changes in human Alzheimer’s disease" was published in 2015. Journal: Alzheimers Res Ther.

Overall, the experimental group should be matched as closely as possible with the controls and the case selection based on the question investigated. The quantitative findings should be controlled for the influences of any *pre-* or *post-mortem* factors or both. Access to detailed clinical records is becoming an important point for the analysis of any quantitative assessment, information which might not be available or which might be incomplete because of the age of the case.

Other factors to account for the analysis are the known genetic risk factors. The polymorphism of the apolipoprotein E (*APOE)* gene is the major risk factor for sporadic AD [16], a fact recently reiterated in a number of genome-wide association studies (GWASs) [17,18]. In the context of inflammation in AD, this is an important point to consider in the constitution of the cohort to study as *APOE* genotype has been associated with microglial activation both in the degree of microglial activation in AD brains [19] and in the microglial expression of inflammatory molecules [20].

## How to analyse the neuroinflammatory response

As mentioned above, different types of tissue are available from brain banks, and the most common are fixed paraffin-embedded and frozen tissue. Fixed paraffin-embedded tissue will be useful to perform immunohistochemical detection of markers of interest. Brain sections could be used at a range of thickness (4 to 30 μm), depending on the experimental needs. The use of thick sections (20 to 30 μm) combined with free-floating immunohistochemistry is highly encouraged (sometimes available if fixed tissue is not paraffin-embedded), as it facilitates the permeation of the antibodies and provides a more effective removal of background staining. Glass-mounted thin sections (4 to 10 μm) can also give good results provided that appropriate protocol optimization is performed. Neuroinflammation can be analyzed in fixed tissue in different but complementary approaches: the qualitative or quantitative assessment or both. Qualitative assessment relies on description according to set criteria and thus can be interpreted as a subjective assessment. Qualitative assessment to be obtained on tissue is (i) the presence or absence of the marker of interest, (ii) the type of cell or feature recognized by the marker, and (iii) the cell morphology (for example, amoeboid, ramified, or dystrophic). However, it is now recognized that morphology is not sufficient to reflect the multitude of functions or activation states expressed by microglia [21]. Therefore, the quantitative approach is essential to obtain an objective measurement of the different markers studied. Quantification relies on sampling and statistical analysis based on numerical data collected. A semi-quantitative analysis can be performed on the basis of a rating system such as a scale of severity/intensity of the marker of interest, defined according to the pattern of immunostaining (for example, 0, 1+, 2+, and 3+) and usually assessed blindly by at least two researchers. Quantitative assessment can be obtained as (i) the number of positive cells per field or per area/volume unit, (ii) the protein load defined as the percentage of the immunostained area of region sampled, and thus (iii) the protein load per cell. For example, Iba1 (ionized calcium-binding adaptor molecule 1) is currently acknowledged as being expressed independently of microglial functional state [22], and its expression is increased during neuroinflammation. Detection of Iba1 is widely used in animal studies, and Iba1 is the reference marker for microglial assessment in the human brain [23]. The numerical data collected are important for statistical power, and collection can be achieved in different ways: (i) by having sufficient cases in each group, (ii) by assessing several brain areas if there are not enough cases, (iii) by collecting enough individual data within each case, or (iv) by doing a combination of these.

The article "Post-mortem analysis of neuroinflammatory changes in human Alzheimer’s disease" was published in 2015. Journal: Alzheimers Res Ther.

The use of frozen tissue will allow the study of gene expression (for example, RT-PCR and microarrays) and protein expression (such as multiplex assays and Western blotting). The RNA or protein isolation methods should match the requirements of the techniques to be applied, and sample size, RNA species, and purity are the main variables to take into account. Owing to the intrinsic value of the human samples, it is highly encouraged when analyzing RNA expression to use isolation kits allowing the purification of all species of RNA, including microRNA, which will allow the multiple analysis. As mentioned previously, quality of frozen tissue is one challenge of *post-mortem* brain; thus, in addition to the parameters described above, adequate experimental controls are essential for the data analysis.

Microglia, as the brain macrophages, have the property to express a range of inflammatory markers [21,24-28]. If the considerations described above are taken into account, functional immune changes can be assessed in the human brain by using specific markers as detailed below.

### Inflammatory profile

Despite a broad interest in the inflammatory response in AD and the extensive research in this disease, the scientific community has failed to shed clear and uniform light on the contribution of local inflammation to the disease [29,30]. The neuropathology of AD shows a robust innate immune response characterized by the presence of activated microglia, with increased or *de novo* expression of diverse macrophage antigens [21], and at least in some cases production of inflammatory cytokines [29,31]. It has been suggested that non-steroidal anti-inflammatory drugs protect from the onset or progression of AD [32], suggesting that inflammation is a causal component of the disease rather than a consequence of the neurodegeneration. Recent GWASs have highlighted several genes involved in innate immunity, indicating also a causal role for inflammation in the disease [33]. Additionally, a solid body of evidence shows that systemic inflammation may interact with the innate immune response in the brain to act as a ‘driver’ of disease progression and exacerbate symptoms [7]. The impact of systemic inflammation on the progression of AD means that any neuropathology study on the inflammatory response in the AD brain must take into account systemic co-morbidities that may influence the microglia phenotype (see ‘Information required for the analysis of the immune response in Alzheimer’s disease’ section).

The definition of the brain inflammatory profile of AD shows conflicting ideas in the literature, probably arising from the heterogeneity of the *post-mortem* samples and the difficult application of the detection methods [21]. AD has been associated with a pro-inflammatory phenotype, characterized by expression of interleukin-1 beta (IL-1β) and complement proteins [34,35]. The upregulation of genes linked to an anti-inflammatory phenotype, arginase 1, or the transforming growth factor-beta (TGF-β) has also been reported in association with AD [36,37]. The consensus defines that, in the human AD brain, the inflammatory response cannot be classified as strictly M1-like or M2-like [38] and that the changes in expression level are compounded by the various detection methods (for review, see [29]).

Although the precise inflammatory phenotype of microglia in AD seems elusive, the link of AD with inflammation seems clear, as highlighted by a recent study using microarray technology on the gene signature of ageing and AD [39]. These ideas support the model of an activation of the innate inflammatory response in microglia as a prelude to the development of AD [39]. Furthermore, studies on incipient AD samples show a strong correlation of genes associated with the microglial response and the progression into AD [40]. The concept of the interconnection of AD and the innate immune response is supported by evidence from a GWAS implicating genes involved in innate immunity [41]. These promising studies are opening new avenues into the understanding of the impact of the innate immune response in AD while supporting the need for future exploration.

The article "Post-mortem analysis of neuroinflammatory changes in human Alzheimer’s disease" was published in 2015. Journal: Alzheimers Res Ther.

Characterising the inflammatory response in human *post-mortem* AD samples by using reliable and consistent methods will provide valuable information in the field. It could be agreed that analysing the expression of inflammatory mediators at the protein level, rather than the analysis of the mRNA expression, is highly desirable. To accomplish this task, the market offers a number of multiplex systems to analyse several molecules simultaneously, accelerating research and minimising costs. It is highly encouraged to analyse a broad range of inflammatory mediators instead of using a limited number of molecules as a proxy. New technical progress aimed at increasing the panel of molecules to be analysed, as well as the detection levels, will provide a valuable approach to be able to trace comparisons like those recently used to define the microglial gene signature in mice [42,43].

### Phagocytosis

The phagocytic ability of microglia is a feature shared with peripheral macrophages, helping to eliminate bacterial, necrotic, or apoptotic cells during development or disease. In AD, the amyloid plaque burden increases with age in both mouse models [44] and human patients [45], indicating the rather ineffective phagocytic potential of microglia. Amyloid-beta (Aβ) deposits have been shown to have a potent chemoattractant activity on microglia, although their removal by phagocytosis has not been clearly evidenced *in vivo* [46]. However, it has been shown that the removal of Aβ can be improved by further challenge of microglia with high doses of lipopolysaccharide [47] or the induction of IL-1β [48]. In human AD, active immunotherapy directed against Aβ has been successful in Aβ removal, partly by redirecting the microglia toward Aβ [23] and by increasing their phagocytic activity [49]. Recent evidence supports a differential contribution of perivascular macrophages and parenchymal microglia, not bone marrow-derived cells, to the clearance of Aβ [50]. In this study, the authors used mice deficient in CCR2, a molecule expressed by monocytes defining their migration, to rule out the contribution of circulating monocytes, further evidencing a prominent role of the perivascular macrophage population to Aβ clearance [50]. Interestingly, as microglia do not express CCR2 in healthy and diseased conditions [51,52], the analysis of this molecule in comparison with other markers expressed by microglia (that is, CX3CR1) can help to potentially differentiate the infiltrated monocytes/macrophages from the resident microglia. This comparison has not been performed yet in the human brain and would provide valuable insights for the understanding of the balance of microglia/macrophages.

The article "Post-mortem analysis of neuroinflammatory changes in human Alzheimer’s disease" was published in 2015. Journal: Alzheimers Res Ther.

The regulation of the phagocytic activity of microglia appears as a key genetic determinant of AD pathology. Recent studies link genetic variants of TREM2, a protein regulating the activation and phagocytic functions of myeloid cells, with the risk of developing AD [53,54]. TREM2 has a balancing role between phagocytic and pro-inflammatory microglial activities and is expressed in microglia around plaques in an experimental model of AD [55]. Similarly, dysregulation of the complement system in humans has been associated with AD [18]. However, no clear consensus defines the overall level of microglial phagocytosis in the human AD brain. The use of refined experimental approaches to directly study microglial phagocytosis [56], together with the analysis of immunological markers such as CD68 (related with phagocytic activity), will shed light on the understanding of the phagocytic activity of microglia and other macrophage populations in the AD brain.

### Proliferation

Microglial activation in neurodegeneration is accompanied by an increase in their numbers. The contribution of circulating progenitors to the microglial population is minor, or even absent, as shown in a mouse model of AD [50], pointing to *in situ* microglial proliferation as the mechanism regulating microglial turnover [57]. In mice, microglia are maintained and function largely independently of circulating progenitors in health [58,59] and disease [50,52,60]. Therefore, the analysis of microglial proliferation in AD is necessary for understanding how the innate inflammatory response contributes to disease onset or progression or both.

Proliferation was assumed to be responsible for the increased number of microglial cells observed in AD samples, although direct evidence of proliferating microglial cells (that is, Ki67 expression in Iba1^+^ cells) was reported only recently [60]. The expansion of the microglial population has been consistently documented in transgenic mouse models of AD, mainly accumulating around plaques [61]. However, direct evidence of microglial proliferation (incorporation of 5-bromo-2-deoxyuridine in Iba1^+^ cells) was only recently reported, suggesting a direct effect of the plaque microenvironment over the regulation of microglial proliferation [62]. These studies pinpoint the importance of the control of microglial proliferation during AD. Establishing reproducible and consistent methods to monitor microglial proliferation in *post-mortem* AD brains will provide the scientific community with valuable tools to better compare results across cohorts of patients, contributing to our better understanding of the pathophysiology of AD [63].

The article "Post-mortem analysis of neuroinflammatory changes in human Alzheimer’s disease" was published in 2015. Journal: Alzheimers Res Ther.

The analysis of microglial proliferation is best achieved by double/triple immunohistochemical analysis by using either fluorescence or bright-field microscopy [63] (Figure 1). The use of fluorescence-based techniques needs to be supplemented by the use of a fluorescence-quenching step (for example, Sudan Black). This step is particularly important in the case of AD human tissue, as the occurrence of autofluorescent artefacts (for example, lipofuscin granules) is very frequent and can compound the interpretation of results. Double bright-field immunohistochemistry can be achieved by combining DAB and alkaline phosphatase reactions, labelling two individual antibodies with a brown or blue precipitate, respectively. Both fluorescent and bright-field microscopy methods need to implement a membrane or cytoplasmic microglial marker (Iba1, CD68, and CD11b) and a nuclear proliferation marker (Ki67, phospho-histone H3, and PCNA), together with nuclear counterstaining to decipher the subcellular localization of the proliferation markers. The analysis of double- or triple-staining techniques needs to be coupled to colour deconvolution methods.

**Figure 1:** **Microglial proliferation in** ***post-mortem*** **human Alzheimer’s disease brain.** Representative images of the detection of Ki67 in microglial cells (Iba1^+^) by bright-field double immunohistochemistry **(A)** (DAB, brown, Iba1; AP, blue, Ki67) or double immunofluorescence **(B)** (Alexa 568, red, Iba1; Alexa 488, green, Ki67) from the temporal cortex of a patient with Alzheimer’s disease. Images adapted from [63]. Iba1, ionized calcium-binding adaptor molecule 1.

### Cell infiltration

Cell infiltration in the brain during AD is an important question related to the potential roles for recruited monocytes/macrophages and T cells within the brain parenchyma. Infiltration of peripheral leukocytes in the human AD brain is very limited when compared with classic autoimmune diseases like multiple sclerosis [64]. However, the rare coincidence of stroke and AD leads to an increase in infiltrating macrophages in the brain, which contained Aβ fibrils suggesting an effective plaque clearance response [65]. Although limited evidence is available in the literature regarding the existence and role of infiltrated leukocytes in human AD, these studies suggest that systemic co-morbidities could determine the degree of infiltration of circulating leukocytes. It should be noted that the findings on analysis of *post-mortem* tissue several years following any event which might impact on neuroinflammation (insult, trauma, disease, treatment) may not necessarily reflect those immediately after the event, and instead represent the later effects.

The article "Post-mortem analysis of neuroinflammatory changes in human Alzheimer’s disease" was published in 2015. Journal: Alzheimers Res Ther.

As explained before (in the ‘Proliferation’ section), experiments in mouse models of AD suggest that the infiltration of circulating monocytes is scarce and does not contribute to the pool of parenchymal microglia [52]. Translating these findings to the human situation is a challenging task because of the lack of specific markers to distinguish microglia from peripheral leukocytes, although the analysis of the levels of molecules like CD45, Ly6C, or CD11c could help to split the contribution from both populations [66].

The study of the adaptive immune response in AD has provided valuable information in the last few years. T-cell number—both the CD4^+^ (T helper) and the CD8^+^ (T cytotoxic/suppressor) populations—increases in patients with AD [67]. Although the number of T cells is higher in AD brains, they do not express markers of proliferation, indicating an absence of antigen-triggered clonal expansion [67]. However, there is evidence indicating the orchestration of a systemic T-cell response, as suggested by the presence of the RO isoform of CD45 in peripheral T cells in patients with AD, linked to T-cell memory [68], and by the increase in the CD4^+^ and CD25^+^ regulatory subsets in patients with AD [69]. However, the role of the T cells infiltrated in the brains of patients with AD is unclear. Major histocompatibility complex class II is found upregulated in microglia surrounding Aβ plaques in the AD brain, indicating possible antigen presentation [30]. However, the co-stimulatory factors CD80 and CD86 are required for the induction of primary adaptive immune responses and their description in microglia in AD remains elusive [70]. Infiltration of T lymphocytes has been associated with the development of side effects in a number of AD patients immunised against Aβ [71,72]. However, analysis of T cells in a cohort of immunised AD cases compared with unimmunised AD cases did not show a difference [23]. Therefore, a detailed analysis of the T cell-dependent responses in the brain parenchyma is required to fully understand the role of these cells in AD pathology. The use of fresh samples, allowing flow cytometry analysis and cell culture [73], would provide the optimal tool to overcome the limitations of using *post-mortem* tissue for this purpose.

The article "Post-mortem analysis of neuroinflammatory changes in human Alzheimer’s disease" was published in 2015. Journal: Alzheimers Res Ther.

## Conclusions

A number of recent publications have highlighted specific inflammatory profiles associated with healthy or diseased brain [38,39]. However, our current knowledge of the neuroinflammatory response in AD is based mainly on *in vitro* and animal studies. Therefore, it is essential to confirm or contradict the experimental findings in the human brain in order to increase our knowledge of the pathogenic mechanisms of AD. This strategy would lead to the identification of potential therapeutic targets without undermining the benefit of animal models. The recent development of brain banks with the aim of providing good-quality tissue for research, in association with the tools now available to identify genes and proteins (Table 1), should soon increase our understanding of the role of immunity in neurodegenerative diseases.

**Table 1:** **Analysis of immune changes in human** ***post-mortem*** **tissue**

Human *post-mortem* tissue	- Genetic heterogeneity
	- Age and gender
	- Agonal status
	- Co-morbidities
	- Cause of death
	- Post-mortem interval
Techniques	
Fixed tissue	- Immunohistochemistry
	○ Bright-field microscopy [23,49,60]
	○ Fluorescent microscopy [23,49,60]
	○ Combination of different markers [23,49,60]
Frozen tissue	- Genomics [39]
	- Proteomics [74]
	- RNA/DNA analysis [38,75,76]
	- Primary culture [73]
	- Flow cytometry [73]
Assessment	
Qualitative	- Cell type
	- Cell morphology
Quantitative	- Semi-quantitative rating system
	- Number of cells per area or volume unit
	- Protein load (percentage)
Immune functions	
Inflammatory profile	- Pro- versus anti-inflammatory cytokines
	- CD14, CD40, major histocompatibility complex II, arginase 1, chitinase, and TREM2
Phagocytosis	- Scavenger receptors (CD68 and CD36), TREM2, FcγRs CD14/TLR4, and phosphatidylserine receptors
Proliferation	- Ki67, PCNA, and phospho-histone H3
Immune cell infiltration	- Monocytes
	○ CCR2 combined with CX3CR1
	○ CD45, LyC6, and CD11c
	- T cells
	○ CD4 (T helper)
	○ CD8 (T cytotoxic/suppressor)

## Note

This article is part of a series on *Innate Immunity*, edited by Donna Wilcock. Other articles in this series can be found at http://alres.com/series/innateimmunity.

## Abbreviations

AD: Alzheimer’s disease
APOE: Apolipoprotein E
Aβ: Amyloid-beta
GWAS: Genome-wide association study
HTA: Human tissue authority
Iba1: Ionized calcium-binding adaptor molecule 1
IL-1β: Interleukin-1 beta
RIN: RNA integrity number
TGF-β: Transforming growth factor-beta

The article "Post-mortem analysis of neuroinflammatory changes in human Alzheimer’s disease" was published in 2015. Journal: Alzheimers Res Ther.

## References

[1] Kasper BS, Taylor DC, Janz D, Kasper EM, Maier M, Williams MR (2010). Neuropathology of epilepsy and psychosis: the contributions of J.A.N. Corsellis. Brain..

[2] Franco R, Cedazo-Minguez A (2014). Successful therapies for Alzheimer’s disease: why so many in animal models and none in humans?. Front Pharmacol..

[3] McCullumsmith RE, Hammond JH, Shan D, Meador-Woodruff JH (2014). Postmortem brain: an underutilized substrate for studying severe mental illness. Neuropsychopharmacology..

[4] Brain Banks in the world [http://wwwbrainnet-europeorg/indexphp?option=com_content&view=article&id=102&Itemid=102]

[5] Norden DM, Godbout JP (2013). Microglia of the aged brain: primed to be activated and resistant to regulation. Neuropathol Appl Neurobiol..

[6] Hynd MR, Lewohl JM, Scott HL, Dodd PR (2003). Biochemical and molecular studies using human autopsy brain tissue. J Neurochem..

[7] Holmes C (2013). Systemic inflammation and Alzheimer’s disease. Neuropathol Appl Neurobiol..

[8] Holmes C, Cunningham C, Zotova E, Woolford J, Dean C, Kerr S (2009). Systemic inflammation and disease progression in Alzheimer disease. Neurology..

[9] Holmes C, El-Okl M, Williams AL, Cunningham C, Wilcockson D, Perry VH (2003). Systemic infection, interleukin 1beta, and cognitive decline in Alzheimer’s disease. J Neurol Neurosurg Psychiatry..

[10] Perry VH, Cunningham C, Holmes C (2007). Systemic infections and inflammation affect chronic neurodegeneration. Nat Rev Immunol..

[11] Cunningham C, Campion S, Lunnon K, Murray CL, Woods JF, Deacon RM (2009). Systemic inflammation induces acute behavioral and cognitive changes and accelerates neurodegenerative disease. Biol Psychiatry..

[12] Burry RW (2011). Controls for immunocytochemistry: an update. J Histochem Cytochem..

[13] Schroeder A, Mueller O, Stocker S, Salowsky R, Leiber M, Gassmann M (2006). The RIN: an RNA integrity number for assigning integrity values to RNA measurements. BMC Mol Biol..

[14] Stan AD, Ghose S, Gao XM, Roberts RC, Lewis-Amezcua K, Hatanpaa KJ (2006). Human postmortem tissue: what quality markers matter?. Brain Res..

[15] Ellis PD (2010). The Essential Guide to Effect Sizes: Statistical Power, Meta-Analysis, and the Interpretation of Research Results.

[16] Genin E, Hannequin D, Wallon D, Sleegers K, Hiltunen M, Combarros O (2011). APOE and Alzheimer disease: a major gene with semi-dominant inheritance. Mol Psychiatry..

[17] Harold D, Abraham R, Hollingworth P, Sims R, Gerrish A, Hamshere ML (2009). Genome-wide association study identifies variants at CLU and PICALM associated with Alzheimer’s disease. Nat Genet..

The article "Post-mortem analysis of neuroinflammatory changes in human Alzheimer’s disease" was published in 2015. Journal: Alzheimers Res Ther.

[18] Lambert JC, Heath S, Even G, Campion D, Sleegers K, Hiltunen M (2009). Genome-wide association study identifies variants at CLU and CR1 associated with Alzheimer’s disease. Nat Genet..

[19] Egensperger R, Kosel S, von Eitzen U, Graeber MB (1998). Microglial activation in Alzheimer disease: association with APOE genotype. Brain Pathol..

[20] Lynch JR, Morgan D, Mance J, Matthew WD, Laskowitz DT (2001). Apolipoprotein E modulates glial activation and the endogenous central nervous system inflammatory response. J Neuroimmunol..

[21] Boche D, Perry VH, Nicoll JA (2013). Activation patterns of microglia and their identification in the human brain. Neuropathol Appl Neurobiol..

[22] Ito D, Imai Y, Ohsawa K, Nakajima K, Fukuuchi Y, Kohsaka S (1998). Microglia-specific localisation of a novel calcium binding protein, Iba1. Brain Res Mol Brain Res..

[23] Zotova E, Bharambe V, Cheaveau M, Morgan W, Holmes C, Harris S (2013). Inflammatory components in human Alzheimer’s disease and after active amyloid-beta42 immunization. Brain..

[24] Gordon S (2003). Alternative activation of macrophages. Nat Rev Immunol..

[25] Lucin KM, Wyss-Coray T (2009). Immune activation in brain aging and neurodegeneration: too much or too little?. Neuron..

[26] Mosser DM, Edwards JP (2008). Exploring the full spectrum of macrophage activation. Nat Rev Immunol..

[27] Colton C, Wilcock DM (2010). Assessing activation states in microglia. CNS Neurol Disord Drug Targets..

[28] Colton CA (2009). Heterogeneity of microglial activation in the innate immune response in the brain. J Neuroimmune Pharmacol..

[29] Ransohoff RM, Perry VH (2009). Microglial physiology: unique stimuli, specialized responses. Annu Rev Immunol..

[30] Akiyama H, Barger S, Barnum S, Bradt B, Bauer J, Cole GM (2000). Inflammation and Alzheimer’s disease. Neurobiol Aging..

[31] Dickson DW, Lee SC, Mattiace LA, Yen SH, Brosnan C (1993). Microglia and cytokines in neurological disease, with special reference to AIDS and Alzheimer’s disease. Glia..

[32] Hoozemans JJ, Veerhuis R, Rozemuller JM, Eikelenboom P (2011). Soothing the inflamed brain: effect of non-steroidal anti-inflammatory drugs on Alzheimer’s disease pathology. CNS Neurol Disord Drug Targets..

[33] Perry VH, Holmes C (2014). Microglial priming in neurodegenerative disease. Nat Rev Neurol..

[34] McGeer PL, Akiyama H, Itagaki S, McGeer EG (1989). Activation of the classical complement pathway in brain tissue of Alzheimer patients. Neurosci Lett..

[35] Griffin WS, Stanley LC, Ling C, White L, MacLeod V, Perrot LJ (1989). Brain interleukin 1 and S-100 immunoreactivity are elevated in Down syndrome and Alzheimer disease. Proc Natl Acad Sci U S A..

The article "Post-mortem analysis of neuroinflammatory changes in human Alzheimer’s disease" was published in 2015. Journal: Alzheimers Res Ther.

[36] Colton CA, Mott RT, Sharpe H, Xu Q, Van Nostrand WE, Vitek MP (2006). Expression profiles for macrophage alternative activation genes in AD and in mouse models of AD. J Neuroinflammation..

[37] Wang G, Zhang Y, Chen B, Cheng J (2003). Preliminary studies on Alzheimer’s disease using cDNA microarrays. Mech Ageing Dev..

[38] Sudduth TL, Schmitt FA, Nelson PT, Wilcock DM (2013). Neuroinflammatory phenotype in early Alzheimer’s disease. Neurobiol Aging..

[39] Cribbs DH, Berchtold NC, Perreau V, Coleman PD, Rogers J, Tenner AJ (2012). Extensive innate immune gene activation accompanies brain aging, increasing vulnerability to cognitive decline and neurodegeneration: a microarray study. J Neuroinflammation..

[40] Blalock EM, Geddes JW, Chen KC, Porter NM, Markesbery WR, Landfield PW (2004). Incipient Alzheimer’s disease: microarray correlation analyses reveal major transcriptional and tumor suppressor responses. Proc Natl Acad Sci U S A..

[41] Jones L, Holmans PA, Hamshere ML, Harold D, Moskvina V, Ivanov D (2010). Genetic evidence implicates the immune system and cholesterol metabolism in the aetiology of Alzheimer’s disease. PLoS One..

[42] Butovsky O, Jedrychowski MP, Moore CS, Cialic R, Lanser AJ, Gabriely G (2014). Identification of a unique TGF-beta-dependent molecular and functional signature in microglia. Nat Neurosci..

[43] Hickman SE, Kingery ND, Ohsumi TK, Borowsky ML, Wang LC, Means TK (2013). The microglial sensome revealed by direct RNA sequencing. Nat Neurosci..

[44] Dodart JC, May P. Overview on rodent models of Alzheimer’s disease. Curr Protoc Neurosci. 2005;Chapter 9:Unit 9.22.10.1002/0471142301.ns0922s3318428631

[45] Okello A, Koivunen J, Edison P, Archer HA, Turkheimer FE, Nagren K (2009). Conversion of amyloid positive and negative MCI to AD over 3 years: an 11C-PIB PET study. Neurology..

[46] Sierra A, Abiega O, Shahraz A, Neumann H (2013). Janus-faced microglia: beneficial and detrimental consequences of microglial phagocytosis. Front Cell Neurosci..

[47] Herber DL, Roth LM, Wilson D, Wilson N, Mason JE, Morgan D (2004). Time-dependent reduction in Abeta levels after intracranial LPS administration in APP transgenic mice. Exp Neurol..

[48] Shaftel SS, Kyrkanides S, Olschowka JA, Miller JN, Johnson RE, O’Banion MK (2007). Sustained hippocampal IL-1 beta overexpression mediates chronic neuroinflammation and ameliorates Alzheimer plaque pathology. J Clin Invest..

[49] Zotova E, Holmes C, Johnston D, Neal JW, Nicoll JA, Boche D (2011). Microglial alterations in human Alzheimer’s disease following Abeta42 immunization. Neuropathol Appl Neurobiol..

The article "Post-mortem analysis of neuroinflammatory changes in human Alzheimer’s disease" was published in 2015. Journal: Alzheimers Res Ther.

[50] Mildner A, Schlevogt B, Kierdorf K, Bottcher C, Erny D, Kummer MP (2011). Distinct and non-redundant roles of microglia and myeloid subsets in mouse models of Alzheimer’s disease. J Neurosci..

[51] Saederup N, Cardona AE, Croft K, Mizutani M, Cotleur AC, Tsou CL (2010). Selective chemokine receptor usage by central nervous system myeloid cells in CCR2-red fluorescent protein knock-in mice. PLoS One..

[52] Gomez-Nicola D, Schetters ST, Perry VH (2014). Differential role of CCR2 in the dynamics of microglia and perivascular macrophages during prion disease. Glia..

[53] Jonsson T, Stefansson H, Steinberg S, Jonsdottir I, Jonsson PV, Snaedal J (2012). Variant of TREM2 associated with the risk of Alzheimer’s disease. N Engl J Med..

[54] Guerreiro R, Wojtas A, Bras J, Carrasquillo MM, Rogaeva E, Majounie E (2012). TREM2 variants in Alzheimer’s disease. N Engl J Med..

[55] Frank S, Burbach GJ, Bonin M, Walter M, Streit W, Bechmann I (2008). TREM2 is upregulated in amyloid plaque-associated microglia in aged APP23 transgenic mice. Glia..

[56] Sierra A, Encinas JM, Deudero JJ, Chancey JH, Enikolopov G, Overstreet-Wadiche LS (2010). Microglia shape adult hippocampal neurogenesis through apoptosis-coupled phagocytosis. Cell Stem Cell..

[57] Gomez-Nicola D, Perry VH. Microglial dynamics and role in the healthy and diseased brain: a paradigm of functional plasticity. Neuroscientist. 2014;21(2):169–184. 10.1177/1073858414530512PMC441287924722525

[58] Ginhoux F, Greter M, Leboeuf M, Nandi S, See P, Gokhan S (2010). Fate mapping analysis reveals that adult microglia derive from primitive macrophages. Science..

[59] Ajami B, Bennett JL, Krieger C, Tetzlaff W, Rossi FM (2007). Local self-renewal can sustain CNS microglia maintenance and function throughout adult life. Nat Neurosci..

[60] Gomez-Nicola D, Fransen NL, Suzzi S, Perry VH (2013). Regulation of microglial proliferation during chronic neurodegeneration. J Neurosci..

[61] Bolmont T, Haiss F, Eicke D, Radde R, Mathis CA, Klunk WE (2008). Dynamics of the microglial/amyloid interaction indicate a role in plaque maintenance. J Neurosci..

[62] Kamphuis W, Orre M, Kooijman L, Dahmen M, Hol EM (2012). Differential cell proliferation in the cortex of the APPswePS1dE9 Alzheimer’s disease mouse model. Glia..

[63] Gomez-Nicola D, Perry VH. Analysis of microglial proliferation in Alzheimer’s disease. Systems biology of Azlheimer’s disease. Methods Mol Biol. in press.10.1007/978-1-4939-2627-5_1026235067

[64] Rezai-Zadeh K, Gate D, Town T (2009). CNS infiltration of peripheral immune cells: D-Day for neurodegenerative disease?. J Neuroimmune Pharmacol..

[65] Wisniewski HM, Barcikowska M, Kida E (1991). Phagocytosis of beta/A4 amyloid fibrils of the neuritic neocortical plaques. Acta Neuropathol (Berl)..

The article "Post-mortem analysis of neuroinflammatory changes in human Alzheimer’s disease" was published in 2015. Journal: Alzheimers Res Ther.

[66] Rose S, Misharin A, Perlman H (2012). A novel Ly6C/Ly6G-based strategy to analyze the mouse splenic myeloid compartment. Cytometry A..

[67] Togo T, Akiyama H, Iseki E, Kondo H, Ikeda K, Kato M (2002). Occurrence of T cells in the brain of Alzheimer’s disease and other neurological diseases. J Neuroimmunol..

[68] Tan J, Town T, Abdullah L, Wu Y, Placzek A, Small B (2002). CD45 isoform alteration in CD4+ T cells as a potential diagnostic marker of Alzheimer’s disease. J Neuroimmunol..

[69] Lombardi VR, Garcia M, Rey L, Cacabelos R (1999). Characterization of cytokine production, screening of lymphocyte subset patterns and in vitro apoptosis in healthy and Alzheimer’s Disease (AD) individuals. J Neuroimmunol..

[70] O’Keefe GM, Nguyen VT, Benveniste EN (2002). Regulation and function of class II major histocompatibility complex, CD40, and B7 expression in macrophages and microglia: implications in neurological diseases. J Neurovirol..

[71] Nicoll JA, Wilkinson D, Holmes C, Steart P, Markham H, Weller RO (2003). Neuropathology of human Alzheimer disease after immunization with amyloid-beta peptide: a case report. Nat Med..

[72] Orgogozo JM, Gilman S, Dartigues JF, Laurent B, Puel M, Kirby LC (2003). Subacute meningoencephalitis in a subset of patients with AD after Abeta42 immunization. Neurology..

[73] Mulder SD, Nielsen HM, Blankenstein MA, Eikelenboom P, Veerhuis R (2014). Apolipoproteins E and J interfere with amyloid-beta uptake by primary human astrocytes and microglia in vitro. Glia..

[74] Lunnon K, Smith R, Hannon E, De Jager PL, Srivastava G, Volta M (2014). Methylomic profiling implicates cortical deregulation of ANK1 in Alzheimer’s disease. Nat Neurosci..

[75] Culpan D, Kehoe PG, Love S (2011). Tumour necrosis factor-alpha (TNF-alpha) and miRNA expression in frontal and temporal neocortex in Alzheimer’s disease and the effect of TNF-alpha on miRNA expression in vitro. Int J Mol Epidemiol Genet..

[76] Culpan D, Cram D, Chalmers K, Cornish A, Palmer L, Palmer J (2009). TNFR-associated factor-2 (TRAF-2) in Alzheimer’s disease. Neurobiol Aging..

